The article "Suppression of microRNA-135b-5p protects against myocardial ischemia/reperfusion injury by activating JAK2/STAT3 signaling pathway in mice during sevoflurane anesthesia" was retracted in 2021. Reasons: duplicated images; signs of a paper mill.

# Suppression of microRNA-135b-5p protects against myocardial ischemia/reperfusion injury by activating JAK2/STAT3 signaling pathway in mice during sevoflurane anesthesia

**DOI:** 10.1042/BSR20170186

**Published:** 2017-06-27

**Authors:** Xiao-Juan Xie, Dong-Mei Fan, Kai Xi, Ya-Wei Chen, Peng-Wei Qi, Qian-Hui Li, Liang Fang, Li-Gang Ma

**Affiliations:** 1 Department of Anesthesiology, The First Affiliated Hospital of Henan University of Science and Technology (New District Hospital), Luoyang 471300, P.R. China; 2 Department of Obstetrics and Gynecology, The First Affiliated Hospital of Henan University of Science and Technology, Luoyang 471300, P.R. China; 3 Department of ENT, The First Affiliated Hospital of Henan University of Science and Technology (New District Hospital), Luoyang 471300, P.R. China; 4 Department of Obstetrics and Gynecology, Luoyang Women and Children's Medical Health Care Center, Luoyang 471300, P.R. China; 5 Department of Anesthesiology, The Second Affiliated Hospital of Henan University of Science and Technology, Luoyang 471300, P.R. China

**Keywords:** Inhalation anesthesia, JAK2/STAT3 signaling pathway, MicroRNA-135b-5p, Myocardial ischemia/reperfusion injury, Sevoflurane

## Abstract

The study aims to explore the effects of *miR-135b-5p* on myocardial ischemia/reperfusion (I/R) injuries by regulating Janus protein tyrosine kinase 2 (JAK2)/signal transducer and activator of transcription (STAT) signaling pathway by mediating inhalation anesthesia with sevoflurane. A sum of 120 healthy Wistar male mice was assigned into six groups. Left ventricular ejection fraction (LVEF) and left ventricular shortening fraction (LVSF) were detected. Cardiomyocyte apoptosis was determined by terminal dexynucleotidyl transferase mediated dUTP-biotin nick end labeling (TUNEL) assay. *MiR-135b-5p* expression, mRNA and protein expression of p-STAT3, p-JAK2, STAT3, JAK2, B-cell lymphoma-2 (Bcl-2) and Bcl-2 associated X protein B (Bax) were detected by quantitative real-time PCR (qRT-PCR) and Western blotting. Target relationship between *miR-135b-5p* and JAK2 was confirmed by dual-luciferase reporter assay. The other five groups exhibited increased cardiomyocyte necrosis, apoptosis, *miR-135b-5p* and Bax expression, mRNA expression of JAK2 and STAT3, and protein expression of p-STAT3 and p-JAK2 compared with the sham group, but showed decreased LVEF, LVFS, and Bcl-2 expression. Compared with the model and AG490 + Sevo groups, the Sevo, inhibitor + Sevo and inhibitor + AG490 + Sevo groups displayed reduced cardiomyocyte necrosis, apoptosis, *miR-135b-5p* and Bax expression, but displayed elevated mRNA expression of JAK2 and STAT3, protein expression of p-STAT3 and p-JAK2, LVEF, LVFS and Bcl-2 expression. Compared with the Sevo and inhibitor + AG490 + Sevo groups, the AG490 + Sevo group showed decreased LVEF, LVFS, Bcl-2 expression, mRNA expressions of JAK2 and STAT3, and protein expressions of p-STAT3 and p-JAK2, but increased cardiomyocyte necrosis, apoptosis, and Bax expressions. *MiR-135b-5p* negatively targetted JAK2. Inhibition of *miR-135b-5p* can protect against myocardial I/R injury by activating JAK2/STAT3 signaling pathway through mediation of inhalation anesthesia with sevoflurane.

The article "Suppression of microRNA-135b-5p protects against myocardial ischemia/reperfusion injury by activating JAK2/STAT3 signaling pathway in mice during sevoflurane anesthesia" was retracted in 2021. Reasons: duplicated images; signs of a paper mill.

## Introduction

Ischemic heart disease is one of the major causes of mortality across the world owing to human cardiovascular diseases [1]. Albeit blood reperfusion is required to restore myocardial oxygen supply and improve biological function of ischemic myocardium, it leads to more serious damage to myocardium after reperfusion compared with pure ischemia, which is termed as myocardial ischemia/reperfusion (I/R) injury [2]. Patients undergoing open-heart surgery are subjected to myocardial I/R injury during operation, which is a significant challenge confronted by modern anesthetic practices [3]. Sevoflurane is a volatile anesthetic and has been demonstrated to exhibit cardioprotective functioning [4]. A large number of reports have indicated that inhalational anesthetics including sevoflurane are able to relieve I/R injury [5,6]. Sevoflurane is extensively applied in clinical practices and basic researches owing to its stable induction and rapid recovery pharmacological properties [7]; and it is a promising treatment to protect against post-I/R injury during perioperation [8]. However, the underlying mechanisms for sevoflurane-regulated cardioprotection are poorly understood [3].

MiRNAs are a sort of small noncoding RNA molecules with approximately 22 nts and are implied in negative regulation of gene expression in a number of physiological processes by binding 3′-UTRs of target genes [9]. Increasing evidence has implicated the role of miRNAs in diverse cardiovascular diseases such as ischemic heart disease [10]. Various miRNAs such as *miR-34a, miR-141*, and *miR-126* have been considered as a regulator of myocardial injury or cardiac repair [11–13]. Furthermore, it has been demonstrated that miRNAs could contribute to myocardial I/R injury by regulation of several key signaling pathways in cell cycle, cell survival as well as cell apoptosis [14]. MiR-135b-5p is a member of miRNA family, yet little evidence is reported for its role in the myocardial I/R injury. The Janus protein tyrosine kinase/signal transducer and activator of transcription (JAK/STAT) signaling pathway transduces cellular signals from the plasma membrane to the nucleus and exerts a crucial role in modulating cardioprotection against I/R injury [15,16]. Importantly, the JAK2/STAT3 signaling pathway has been indicated to protect against myocardial I/R injury [17]. Activated p-STAT3 and p-JAK are sufficient enough to prevent cardiomyocyte apoptosis *in vivo* and *in vitro* [18]. However, whether the JAK2/STAT3 pathway participates in the *miR-135b-5p*-mediated reduction in I/R injury has not been clarified. Thus, our study aims to investigate the effects of *miR-135b-5p* on myocardial I/R injury by regulating JAK2/STAT3 signaling pathway through inhalation anesthesia with sevoflurane.

The article "Suppression of microRNA-135b-5p protects against myocardial ischemia/reperfusion injury by activating JAK2/STAT3 signaling pathway in mice during sevoflurane anesthesia" was retracted in 2021. Reasons: duplicated images; signs of a paper mill.

## Materials and methods

### Ethics statement

The study was approved by Animal Ethics Committee, and was in conformity with animal protection, welfare and ethical principles as well as National regulations on animal welfare and ethics.

### Animal grouping and myocardial I/R mice model establishment

A total of 120 healthy Wistar male mice of similar age (weighing 18–22 g) were obtained (Laboratory Animal Center, Academy of Military Medical Sciences of People’s Liberation Army of China, Beijing, China), amongst which 100 mice were randomly selected for myocardial I/R mice model establishment and received 2% pentobarbital sodium intraperitoneal injections (50 mg/ml, batch no. WS20051129; Sinopharm Chemical Reagent Co., Ltd., Shanghai, China). Next, electrocardiogram (ECG) monitoring electrodes were connected to the mice limbs. The small animal ventilator was interiorly aired and applied to the mice with a respiratory frequency of 60 per min and tidal volume of 13–15 ml. The mice underwent thoracotomy at the fourth intercostal space, damage-free stitching and absorbable suture 6-0, which crossed the anterior descending branch of left coronary artery to block the blood vessels. The elevated ST ECG segments signified a successful block. After 30 min, the stitches were loosened to dredge the blood vessels. The resulting reduced ST segments revealed the success of myocardial I/R mice model establishment. The mice contained were randomly classified into six groups based on the randomized table, with 20 mice in each group. The sham group contained mice stitched with damage free and absorbable suture 6-0, which crossed the anterior descending branch of left coronary artery after thoracotomy, yet their blood vessels were not blocked. The model group contained 20 randomly selected myocardial I/R mice deprived of any other treatment. The Sevo group contained 20 randomly selected I/R mice which inhaled 2.8% sevoflurane (batch no. 5X141; Abbott Laboratories, Chicago, IL, U.S.A.) immediately lasting for 5 min after 30-min ischemia and then conducted with reperfusion for 120 min again. The AG490 + Sevo group contained 20 randomly selected I/R mice intravenously injected with AG490 (3 μg/g, JAK enzyme inhibitors and signaling pathway blockers (HY-12000, Sigma–Aldrich Chemical Company, St. Louis, MO, U.S.A.) 5 min before reperfusion and other treatment received were similar to the Sevo group. As for the inhibitor + Sevo group, 20 randomly selected I/R mice intramyocardially injected with *miR-135b-5p* inhibitor (0.2 μl/g, Shanghai GenePharma Co., Ltd., Shanghai, China) 24 h before I/R and other treatment received were similar to the Sevo group 24 h later after chest closure. And for the inhibitor + AG490 + Sevo group, 20 randomly selected I/R mice intramyocardially injected with *miR-135b-5p* inhibitor (0.2 μl/g) 24 h before I/R and intravenously injected with AG490 (3 μg/g) 5 min before reperfusion and other treatment received were just the same as the Sevo group.

The article "Suppression of microRNA-135b-5p protects against myocardial ischemia/reperfusion injury by activating JAK2/STAT3 signaling pathway in mice during sevoflurane anesthesia" was retracted in 2021. Reasons: duplicated images; signs of a paper mill.

### Transthoracic echocardiography

The mice received 2% pentobarbital sodium (WS20051129, Sinopharm Chemical Reagent Co., Ltd., Shanghai, China) intraperitoneal injections and underwent transthoracic echocardiography analyses at T_0_ (30 min prior to ischemia), T_1_ (30 min of ischemia) and T_2_ (120 min of reperfusion). High frequency ultrasonoscope Acuson sequoia 512 (Acuson Corp., Silicon Valley, CA, U.S.A.) was employed at a probe frequency of 8.5 mHz and a scanning speed at 100 mm/s. The mice were anesthetized using 2% pentobarbital sodium and subsequently fixed on the experiment table. The M-curve was measured at the long axis of papillary muscle and left ventricle section level. The following variables were measured and averaged during the three consecutive cardiac cycles: left ventricular end-systolic diameter (LVSD), left ventricular end-diastolic diameter (LVDD), left ventricular end-systolic volume (LVSV), and left ventricular end-diastolic volume (LVDV). The left ventricular ejection fraction (LVEF) and left ventricular fractional shortening (LVFS) values were converted by the Simpson method using the following formula: LVEF = (LVDV – LVSV)/LVDV × 100%; LVFS = (LVDD – LVSD)/LVDD × 100%. LVEF and LVFS were used as parameters indicating cardiac function. The experiment was conducted three times and the mean value was obtained.

### Hematoxylin-eosin staining

Myocardial tissues were fixed with 4% formaldehyde (volume percentage) for 6 h and embedded in impregnated paraffin wax. The tissues were consequently sliced into 3-μm thick sections. The slices were baked overnight at 60°C and dewaxed for 20 min in xylene I and for another 20 min in xylene II. The sections were treated in 100, 90, 80, and 70% ethanol for 5 min, respectively, followed by addition of distilled water. The sections were stained for 10 min using hematoxylin and washed for 15 min to restore blue coloration. Next, the sections were stained for 30 s using eosin, and the red coloration was washed off using double distilled water. Subsequently, the sections were dehydrated, transparentized, and sealed using alcohol, dimethyl benzene, and neutral balsam, respectively. Histopathological examination was conducted by hematoxylin-eosin (HE) staining, myocardial tissue staining as well as the distribution range and staining intensity were also observed. Under 100-times of amplification, morphological image analysis system was applied in order to observe necrosis and edema in myocardial tissues. The images were randomly obtained and the experiment was conducted three times.

The article "Suppression of microRNA-135b-5p protects against myocardial ischemia/reperfusion injury by activating JAK2/STAT3 signaling pathway in mice during sevoflurane anesthesia" was retracted in 2021. Reasons: duplicated images; signs of a paper mill.

### Terminal dexynucleotidyl transferase mediated dUTP-biotin nick end labeling assay

Mice myocardial tissues of each group were fixed with 4% polyformaldehyde, conventionally dehydrated, embedded in paraffin, and sliced into 3-μm thick sections. The sections were subsequently adhered on to polylysine-attached slides, baked for 1 h at 65°C, and were dewaxed and rehydrated. The electric rice cooker being used was filled up with an appropriate amount of water (water depth 3 cm to the plastic dyeing vat), and was subsequently boiled. The sections were placed on to a plastic dyeing rack and submerged in the dyeing vat containing a citric acid buffer of 0.01 mol/l (pH =6.0). Subsequently, the vat was placed in a pot and boiled for 10 min. Once the power was switched off, the vat was insulated for 20 min before it was taken out to cool at room temperature. Next, the sections were washed with PBS, and DNA segments were marked. The following operation was in conformity with instructions of the terminal dexynucleotidyl transferase mediated dUTP-biotin nick end labeling (TUNEL) kit (Nippon Boehringer Ingelheim Co. Ltd., Beijing, China). Observations revealed that the number of the apoptotic nuclei and total cells in each high magnified view, with the addition of six high magnified views of each section. The apoptotic index (AI) referred to the number of apoptotic nucleus amongst 100 nuclei. The average was converted according to the following formula: AI = positive cell number/total cells × 100%. The experiment was repeated three times and the mean value was calculated.

### Quantitative real-time PCR

The total RNA of tissue samples were extracted using a one-step method according to the TRIzol reagent instructions (Invitrogen Inc., Carlsbad, CA, U.S.A.). The RNA at that point was dissolved in ultrapure water treated with diethylpyrocarbonate (Shanghai Sangon Biotech Co., Ltd., Shanghai, China). Absorbance was assessed at wavelengths of 260 and 280 nm with the help of ND-1000 ultraviolet-visible spectrophotometer (Thermo Fisher Scientific, CA, U.S.A.). Total RNA quality was assessed and RNA concentration was adjusted. The extracted RNA was reverse transcribed by a two-step method based on the reagent kit instructions (Thermo Fisher Scientific, CA, U.S.A.). The reaction conditions were as follows: 70°C for 10 min, ice bath for 2 min, 42°C for 60 min, and 70°C for 10 min. The transcribed cDNA was temporarily stored in a refrigerator at –80°C. The quantitative real-time PCR (qRT-PCR) was conducted by the TaqMan probe method, and the reaction was performed according to the reagent kit instructions (MBI Fermentas, Vilnius, Lithuania). The primer sequences are listed in Table 1. The reaction conditions were as follows: 40 cycles of predenaturation at 95°C for 30 s, denaturation at 95°C for 10 s, annealing at 60°C for 20 s, and extension at 70°C for 10 min. The reaction system contained: 12.5 μl of Premix Ex Taq or SYBR Green Mix, 1 μl of forward primer, 1 μl of reverse primer, 1–4 μl of DNA template, and 25 μl of ddH_2_O. The qRT-PCR instrument (Bio–Rad iQ5; Bio–Rad Laboratories, Hercules, CA, U.S.A.) was employed. U6 was used as the internal reference for *miR-135b-5p* [19], and β-actin was used as the internal reference for other target genes. Relative quantitative method was used for calculations and the relative expression of each target gene was presented as 2^−ΔΔ*C*^_t_. The experiment was conducted three times and the mean value was obtained.

The article "Suppression of microRNA-135b-5p protects against myocardial ischemia/reperfusion injury by activating JAK2/STAT3 signaling pathway in mice during sevoflurane anesthesia" was retracted in 2021. Reasons: duplicated images; signs of a paper mill.

**Table 1:** Primer sequences of genes for qRT-PCR

Gene	Sequence
*miR-135b-5p*	Forward: 5′-GCGGCGGTATGGCTTTTCATTC-3′
	Reverse: 5′-ATCCAGTGCAGGGTCCGAGG-3′
*U6*	Forward: 5′-CTCGCTTCGGCAGCACA-3′
	Reverse: 5′-AACGCTTCACGAATTTGCGT-3′
*JAK2*	Forward: 5′-GGTTCATTCAGCAGTTCAGTC-3′
	Reverse: 5′-GCAGGGTCTCCAGGTTTATG-3′
*STAT3*	Forward: 5′-TACCACAAAAGTCAGGTTGCTG-3′
	Reverse: 5′- ACATCCCCAGAGTCCTTATCAA-3′
*Bax*	Forward: 5′-CATCCAGGATCGAGCAGAGAG-3′
	Reverse: 5′-AGCGTAGAAGAGGGCAACC-3′
*Bcl-2*	Forward: 5′-CTACGACTCGGATACTGGAG-3′
	Reverse: 5′-GACAGCCAGGAGAAATCAAAC-3′
*β-actin*	Forward: 5′-GTGCTATGTTGCTCTAGACTTCG-3′
	Reverse: 5′-ATGCCACAGGATTCCATACC-3′

Abbreviations: Bax, Bcl-2 associated X protein B; Bcl-2, B-cell lymphoma-2.

### Western blotting

SDS lysis buffer (1×) was added to the total protein sample. The protein extract was heated at 100°C for 5 min. Supernatant (20 μl) was obtained and electrophoresed in 12% polyacrylamide gel. Once the membrane was formed, it was sealed in a decolorized table at room temperature with tris-buffered saline Tween-20 (TBST) containing 5% BSA. The sealing solution was discarded and the membrane was transferred into a plastic groove. Then, 5% BSA was added to prepare the corresponding concentration of the primary mouse antibody p-STAT3 (1:1000, ab32143), mouse antibody p-JAK2 (1:1000 ab195055), mouse antibody STAT3 (1:1000, ab30647), mouse antibody JAK2 (1:1000, ab195055), mouse antibody Bax (1:1000, ab32503), mouse antibody Bcl-2 (1:1000, ab59348), and mouse antibody β-actin (1:1000, ab195055). All antibodies listed above were purchased from Abcam Inc. (Cambridge, MA, U.S.A.). The membrane was oscillated in the refrigerator with the transfer side facing up at 4°C overnight. The membrane was rinsed with TBST three times with each time for 10 min the following day. The diluted secondary antibody (ab6789; Abcam Inc., Cambridge, MA, U.S.A.) was added and incubated at 4°C for 4–6 h. The membrane at that point was washed with TBST three times (10 min per time). Chemiluminescence reagents A and B solution (Shanghai Yanhui Industrial Co., Ltd., Shanghai, China) were mixed in a ratio of 1:1, and the mixture was dripped on to a nitrocellulose filter membrane. Consequently, the images were obtained after the application of an imaging solution. All Western blotting bands were analyzed in order to obtain relative optical density values. The experiment was conducted three times and the mean value was obtained.

The article "Suppression of microRNA-135b-5p protects against myocardial ischemia/reperfusion injury by activating JAK2/STAT3 signaling pathway in mice during sevoflurane anesthesia" was retracted in 2021. Reasons: duplicated images; signs of a paper mill.

### Cell culture and grouping

Ten mice were randomly selected from each group. The selected mice were killed after disinfection. The thorax was opened quickly and the heart was taken out. The great vessels were cut off from the heart, which was washed and cut into 1 mm chunks. Furthermore, 0.1% trypsin was added for digestion at 37°C for 10 min, and the supernatant was absorbed. The digestion was terminated by Dulbecco’s modified Eagle’s medium (DMEM) (Gibco Company, Grand Island, NY, U.S.A.) containing 10% BSA (Gibco Company, Grand Island, NY, U.S.A.). Next, the heart tissues were centrifuged at a rate of 1000 rpm for 10 min, and consequently, the supernatant was discarded. The DMEM was suspended and the treatment was repeated until complete digestion was observed. Entire cell suspension was collected. Cell density was adjusted to 5 × 10 cells/ml and seeded into a culture bottle or culture plate with a coverslip at the bottom. The tissues were cultured in an incubator and the culture solution was replaced every 2–3 days. The third-generation cells were selected and assigned into the sham group (cells separated from myocardial tissues of mice in the sham group), the model group (cells separated from myocardial tissues of mice in the model group), the Sevo group (cells extracted from myocardial tissues of mice in the Sevo group), the AG490 + Sevo group (cells separated from myocardial tissues of mice in the AG490 + Sevo group), the inhibitor + Sevo group (cells separated from myocardial tissues of mice in the inhibitor + Sevo group), and the inhibitor + AG490 + Sevo group (cells separated from myocardial tissues of mice in the inhibitor + AG490 + Sevo group). The experiment was conducted three times.

The article "Suppression of microRNA-135b-5p protects against myocardial ischemia/reperfusion injury by activating JAK2/STAT3 signaling pathway in mice during sevoflurane anesthesia" was retracted in 2021. Reasons: duplicated images; signs of a paper mill.

### Dual-luciferase reporter assay

MicroRNA.org prediction website was used to analyze the possible target gene of *miR-135b-5p*, and the related segment sequence was obtained accordingly. Cardiomyocyte DNA was extracted based on the instructions of the TIANamp Genomic DNA Kit (TIANGEN Biotech Co., Ltd., Beijing, China). The JAK2 3′-UTR wild-type (wt), JAK2-3′-UTR-wt and mutation type (mut), JAK2-3′-UTR-mut were designed in which *miR-135b-5p* binding region was lost. A luciferase reporter vector was constructed. The *miR-135b-5p* mimics were transfected into cardiomyocytes. The sequence for *miR-135b-5p* mimics was as follows: 5′-UAUGGCUUUUUAUUCCUAUGUGA-3′. Sample luciferase activities were detected in accordance with a luciferase reporter assay kit (Promega Corp., Madison, Wisconsin, U.S.A.). After 48 h of transfection, the residual medium was absorbed and washed twice with PBS. One hundred microliters of passive lysis buffer (PLB) was added to each well. The cell lysate was collected after 15 min of gentle oscillation. The pre-reading time of the program was set at 2 s and reading at 10 s. The sample size of LARIIStop&Glo® Reagent (Promega Corp., Madison, Wisconsin, U.S.A.) was 100 μl. The prepared reagent was placed into light emitting diodes or plates (each sample was 20 μl), and subsequently placed into a chemiluminescence detector (Modulus™; Turner BioSystems, Sunnyvale, CA, U.S.A.). The strongest luciferase intensity was presented at 560 nm wavelength. The experiment was conducted three times and the mean value was obtained.

### Statistical analysis

Statistical analysis was performed using the SPSS 21.0 software (SPSS Inc., Chicago, IL, U.S.A.). Measurement data were demonstrated by mean ± S.D. Differences between multiple groups were compared by one-way ANOVA, and differences between the two groups were compared by *t* test. *P*<0.05 was considered statistically significant.

## Results

### Identification of myocardial I/R injury mouse model

The model group exhibited elevated ST ECG segments postoperation compared with preoperation. After reperfusion, ST segment flattened. No significant change was observed in the sham group during preoperation, intraoperation, and postoperation periods. The results revealed that an anterior descending coronary artery block affected cardiac electrophysiology, and reperfusion restored its functioning. Individual thoracotomy failed to affect cardiac electrophysiology. In addition, the myocardial I/R injury mouse model was successfully established (Figure 1).

The article "Suppression of microRNA-135b-5p protects against myocardial ischemia/reperfusion injury by activating JAK2/STAT3 signaling pathway in mice during sevoflurane anesthesia" was retracted in 2021. Reasons: duplicated images; signs of a paper mill.

**Figure 1:** ECG of the mice in the sham and model group.

### The changes of LVEF and LVFS at T_0_, T_1_, and T_2_ in each group

There were no significant differences in LVEF and LVFS at T_0_ and T_1_ time-periods amongst each group (all *P*>0.05). The LVEF and LVFS at T_2_ amongst the model, Sevo, AG490 + Sevo, inhibitor + Sevo, and inhibitor + AG490 + Sevo groups were significantly different compared with T_0_ time periods (all *P*<0.05). Compared with the sham group, the other five groups displayed reduced LVEF and LVFS at T_2_ time-periods (all *P*<0.05). Compared with the model group, the Sevo, inhibitor + Sevo, and inhibitor + AG490 + Sevo groups showed elevated LVEF and LVFS 120 min after reperfusion (all *P*<0.05), whereas no statistical difference was found in the AG490 + Sevo group (both *P*>0.05). Compared with the Sevo group, AG490 + Sevo group showed declined LVEF and LVFS 120 min after reperfusion (both *P*<0.05). However the inhibitor + Sevo group showed an increment (both *P*<0.05). No significant difference was indicated between the Sevo group and inhibitor + AG490 + Sevo group (both *P*>0.05). Compared with the inhibitor + Sevo group, the LVEF and LVFS were reduced 120 min after reperfusion in the inhibitor + AG490 + Sevo group (both *P*<0.05, Table 2). The experiment was performed on surviving mice devoid of ventricular aneurysm.

**Table 2:** Comparisons of LVEF and LVFS at different time points in mice among each group (*n*=20)

Group	LVEF (%)			LVES (%)		
	T_0_	T_1_	T_2_	T_0_	T_1_	T_2_
Sham	82.52 ± 2.67	81.32 ± 2.55	82.43 ± 2.52	45.52 ± 4.67	45.32 ± 4.55	45.43 ± 3.52
Model	82.36 ± 2.34	83.21 ± 1.12	54.76 ± 1.03^1,*^	45.43 ± 2.34	44.21 ± 1.12	24.76 ± 1.03^1,*^
Sevo	82.32 ± 2.04	83.54 ± 1.96	75.54 ± 1.34^1,2,*^	46.22 ± 2.04	47.54 ± 1.96	35.54 ± 1.34^1,2,*^
AG490 + Sevo	83.02 ± 2.12	84.12 ± 1.34	55.34 ± 1.02^1,3,*^	45.22 ± 2.12	44.12 ± 1.34	26.34 ± 1.02^1,3,*^
Inhibitors + Sevo	82.23 ± 2.34	81.34 ± 2.01	80.21 ± 1.34^1,2,3,*^	46.23 ± 2.34	45.34 ± 2.01	40.21 ± 1.34^1,2,3,*^
Inhibitors + AG490 + Sevo	82.67 ± 2.45	83.97 ± 1.96	74.78 ± 1.24^1,2,4,*^	45.67 ± 2.45	43.97 ± 1.96	36.78 ± 1.24^1,2,4,*^

Abbreviations: LVFS, left ventricular fractional shortening. T_0_, 30 min before ischemia; T_1_, 30 min of ischemia; T_2_, 120 min of reperfusion. ^1^, *P*<0.05 compared with the sham group; ^2^, *P*<0.05 compared with the model group; ^3^, *P*<0.05 compared with the Sevo group; ^4^, *P*<0.05 compared with the inhibitors + Sevo group; *, compared with the T_0_, *P*<0.05; sham, mice with no model establishment; model, mice model with no other treatment; Sevo, mice model treated with sevoflurane injection; AG490 + Sevo, mice model treated with AG490 and sevoflurane injection; inhibitors + Sevo, mice model treated with *miR-135b-5p* inhibitor and sevoflurane injection; inhibitors + AG490 + Sevo groups, mice model treated with *miR-135b-5p*, inhibitor, AG490 and sevoflurane injection.

The article "Suppression of microRNA-135b-5p protects against myocardial ischemia/reperfusion injury by activating JAK2/STAT3 signaling pathway in mice during sevoflurane anesthesia" was retracted in 2021. Reasons: duplicated images; signs of a paper mill.

### Pathological changes of myocardial tissues in each group by HE staining

The sham group displayed orderly and neat myocardial fibers in fascicular fashion under an optical microscope. Additionally, cardiomyocytes presented normal form lacking intercellular edema, orderly and neat stripes, and the caryotheca was intact with uniformly distributed chromatin. Compared with the sham group, the model group displayed disordered myocardial fibers, swelling, significant edema, blurred intercellular boundaries, disappeared striations and extensive cardiomyocyte necrosis. Compared with the model group, the AG490 + Sevo group displayed relatively ordered fibers and reduced necrosis. Moreover, in comparison with the Sevo group, the AG490 + Sevo group displayed disordered fibers, increased cardiomyocyte necrosis, and the inhibitor + Sevo group displayed neat fiber arrays, slight edema, and decreased cardiomyocyte necrosis. Compared with the inhibitor + Sevo group, the inhibitor + AG490 + Sevo group displayed disordered fibers and increased cardiomyocyte necrosis (Figure 2).

**Figure 2:** Histopathological changes in myocardial tissues detected by HE staining in each group (×100) Sham, mice with no model establishment; model, mice model with no other treatment; Sevo, mice model treated with evoflurane injection; AG490 + Sevo, mice model treated with AG490 and sevoflurane injection; inhibitor + Sevo, mice model treated with *miR-135b-5p* inhibitor and sevoflurane injection; inhibitor + AG490 + Sevo groups, mice model treated with *miR-135b-5p*, inhibitor, AG490 and sevoflurane injection.

### Inhibition of *miR-135b-5p* reduced the cardiomyocyte apoptosis in mice suffering from myocardial I/R injury

Presence of apoptotic cells can be seen as the brownish-yellow particles in the nucleus. The sham group was devoid of apoptotic cells. The other five groups displayed an increased amount of apoptotic cells in comparison with the sham group (*P*<0.05). The Sevo, inhibitor + Sevo, and inhibitor + AG490 + Sevo groups displayed significantly reduced cardiomyocyte apoptosis in comparison with the model group (all *P*<0.05), and moreover, no statistical difference was observed in the AG490 + Sevo group (*P*>0.05). The AG490 + Sevo group showed an increase in cardiomyocyte apoptosis compared with the Sevo group (*P*<0.05), but a reduction in the inhibitor + Sevo group (*P*<0.05), whereas no significant difference was indicated in the inhibitor + AG490 + Sevo group (*P*>0.05). The inhibitor + AG490 + Sevo group displayed higher levels of cardiomyocyte apoptosis compared with the inhibitor + Sevo group (*P*<0.05, Figure 3).

The article "Suppression of microRNA-135b-5p protects against myocardial ischemia/reperfusion injury by activating JAK2/STAT3 signaling pathway in mice during sevoflurane anesthesia" was retracted in 2021. Reasons: duplicated images; signs of a paper mill.

**Figure 3:** Cardiomyocyte apoptosis of mice among the six groups (x400) (**A**) TUNEL staining images of cardiomyocyte apoptosis in mice among six groups; (**B**) histogram of AI among six groups; ^a^, compared with the sham group, *P*<0.05; ^b^, compared with the model group, *P*<0.05; ^c^, compared with the Sevo group, *P*<0.05; sham, mice with no model establishment; model, mice model with no other treatment; Sevo, mice model treated with evoflurane injection; AG490 + Sevo, mice model treated with AG490 and sevoflurane injection; inhibitor + Sevo, mice model treated with *miR-135b-5p* inhibitor and sevoflurane injection; inhibitor + AG490 + Sevo groups, mice model treated with *miR-135b-5p*, inhibitor, AG490 and sevoflurane injection.

### MiR-135b-5p expression, mRNA and protein expression of Bcl-2 and Bax of cells and tissues of mice in each group

The other five groups demonstrated elevated *miR-135b-5p* expression and *Bax* mRNA and protein expression as well as an elevated *Bcl-2* mRNA and protein expression compared with the sham group (all *P*<0.05). The Sevo, inhibitor + Sevo and inhibitor + AG490 + Sevo groups showed decreased *miR-135b-5p* expression and mRNA and protein expression of Bax, but an increased mRNA and protein expression of Bcl-2 compared with the model group (all *P*<0.05), the AG490 + Sevo group showed decreased *miR-135b-5p* expression (*P*<0.05) but no significance in mRNA and protein expression of Bax and Bcl-2 (*P*>0.05). The Sevo and the AG490 + Sevo group showed no differences among* miR-135b-5p* expression (*P*>0.05) but the latter group showed an increased mRNA and protein expressions of Bax and decreased Bcl-2 mRNA and protein expression (all *P*<0.05), while the inhibitor + Sevo group exhibited lower *miR-135b-5p* expression and mRNA and protein expression of Bax, and higher mRNA and protein expression of Bcl-2 (all *P*<0.05). The inhibitor + AG490 + Sevo group showed decreased *miR-135b-5p* expression (*P*<0.05) but no significant differences were observed among the mRNA and protein expression of Bax and Bcl-2 (all *P*>0.05). The inhibitor + AG490 + Sevo groups showed no significant differences among *miR-135b-5p* expression when compared with the inhibitor + Sevo group, but showed significantly increased mRNA and protein expression of Bax, and decreased mRNA and protein expression of Bcl-2 (all *P*<0.05, Figure 4).

The article "Suppression of microRNA-135b-5p protects against myocardial ischemia/reperfusion injury by activating JAK2/STAT3 signaling pathway in mice during sevoflurane anesthesia" was retracted in 2021. Reasons: duplicated images; signs of a paper mill.

**Figure 4:** miR-135b-5p expression and mRNA and protein expressions of Bax and Bcl-2 in myocardial tissues and cardiomyocytes among each group. (**A**) Histogram of *miR-135b-5p* expression in myocardial tissues in each group; (**B**) mRNA expressions of Bcl-2 and Bax in myocardial tissues among each group; **C**) Western blotting images and histogram of protein expressions of Bcl-2 and Bax in myocardial tissues among each group. ^a^, compared with the sham group, *P*<0.05; ^b^, compared with the model group, *P*<0.05; ^c^, compared with the Sevo group, *P*<0.05; sham, mice with no model establishment; model, mice model with no other treatment; Sevo, mice model treated with sevoflurane injection; AG490 + Sevo, mice model treated with AG490 and sevoflurane injection; inhibitor + Sevo, mice model treated with *miR-135b-5p* inhibitor and sevoflurane injection; inhibitor + AG490 + Sevo groups, mice model treated with miR-135b-5p, inhibitor, AG490 and sevoflurane injection.

### Inhibition of *miR-135b-5p* increased mRNA expression of JAK2 and STAT3 and protein expression of p-STAT3 and p-JAK2 in mice suffering from myocardial I/R injury

The other five groups demonstrated elevated mRNA and phosphorylated protein expression of JAK2/STAT3 signaling pathway related proteins compared with the sham group (all *P*<0.05). The Sevo, inhibitor + Sevo and inhibitor + AG490 + Sevo groups displayed elevated mRNA expression of JAK2 and STAT3 and protein expression of p-JAK2 and p-STAT3 compared with the sham group (all *P*<0.05), and no significant difference was found in the AG490 + Sevo group (all *P*>0.05). Whereas, the AG490 + Sevo group displayed lower mRNA expression of JAK2 and STAT3 and protein expression of p-JAK2 and p-STAT3 compared with the Sevo group (all *P*<0.05), while the inhibitor + Sevo group presented higher mRNA expression of JAK2 and STAT3 and protein expression of p-JAK2 and p-STAT3 (all *P*<0.05). There was no significant difference between the Sevo and inhibitor + AG490 + Sevo groups (all *P*>0.05). The inhibitor + AG490 + Sevo group displayed lower mRNA expression of JAK2 and STAT3 and protein expression of p-JAK2 and p-STAT3 compared with the inhibitor + Sevo group (all *P*<0.05, Figure 5).

**Figure 5:** mRNA and protein expressions of the JAK2/STAT3 signaling pathway-related proteins in myocardial tissues and cardiomyocytes among each group. (**A**) Histogram of mRNA expressions of JAK2 and STAT3 in myocardial tissues among each group; (**B**) Western blotting images and histogram of protein expressions of p-JAK2 and p-STAT3 in myocardial tissues among each group. ^a^, compared with the sham group, *P*<0.05; ^b^, compared with the model group, *P*<0.05; ^c^, compared with the Sevo group, *P*<0.05; sham, mice with no model establishment; model, mice model with no other treatment; Sevo, mice model treated with evoflurane injection; AG490 + Sevo, mice model treated with AG490 and sevoflurane injection; inhibitor + Sevo, mice model treated with *miR-135b-5p* inhibitor and sevoflurane injection; inhibitor + AG490 + Sevo groups, mice model treated with *miR-135b-5p*, inhibitor, AG490 and sevoflurane injection.

The article "Suppression of microRNA-135b-5p protects against myocardial ischemia/reperfusion injury by activating JAK2/STAT3 signaling pathway in mice during sevoflurane anesthesia" was retracted in 2021. Reasons: duplicated images; signs of a paper mill.

### MiR-135b-5p negatively targetted JAK2

Online software analysis revealed that there was a specific binding region between JAK2 3′-UTR 864–871 sequence and *miR-135b-5p* sequence. JAK2 was the target gene of miR-135b-5p (Figure 6A). Luciferase reporter assay confirmed that *miR-135b-5p* mimics decreased luciferase intensity in the JAK2-3′-UTR-mut group (*P*<0.05) but exerted no significant effects on the luciferase viability in the JAK2-3′-UTR-mut group (*P*>0.05, Figure 6B). The results indicated that *miR-135b-5p* was capable of specifically binding with JAK2-3′-UTR and down-regulating JAK2 expression after transcription.

**Figure 6:** Verification of targeting relationship between miR-135B-5P and JAK2. ^a^, compared with the NC group, *P*<0.05; (**A**) binding region of *miR-135b-5p* on JAK2 3′-UTR; (**B**) histogram of luciferase activity of JAK2-wt and JAK2-mut.

## Discussion

Myocardial I/R injury is a major cause of cardiac dysfunction as well as mortality and morbidity following heart infarctions and cardiac operations [20]. In the present study, we investigated correlations between *miR-135b-5p* and JAK2/STAT3 signaling pathway and their co-functions in myocardial I/R injury, whereby *miR-135b-5p* may mediate inhalation anesthesia with sevoflurane. We found that *miR-135b-5p* inhibition provides protection against myocardial I/R injury by up-regulating JAK2 expression and activating JAK2/STAT3 signaling pathway.

First, we confirmed that sevoflurane could relieve I/R injury and exhibit cardioprotective functioning. The Sevo, inhibitor + Sevo, and inhibitor + AG490 + Sevo groups displayed reduced cardiomyocyte necrosis and apoptosis compared with the model and AG490 + Sevo groups. Inhalational anesthetic of sevoflurane is frequently employed in clinical treatment owing to its stable induction and rapid recovery properties [6], and sevoflurane has been reportedly protective against cardiac injuries [4]. Yang et al. [7] reported that sevoflurane postconditioning might be correlated to mitochondrial respiratory function enhancement and myocardial I/R injury reduction after up-regulation of HIF-1α expression. The findings of Cao et al. [21] indicate that sevoflurane protects myocardial tissues from I/R injury and attenuates the myocardial infarct size by inhibiting the opening of mitochondrial permeability transition pore and reducing extensive autophagy and apoptosis of cardiomyocytes, which are regulated by an increase in NOS as well as the reduction in p-Na^+^/H^+^ exchanger 1 level.

The article "Suppression of microRNA-135b-5p protects against myocardial ischemia/reperfusion injury by activating JAK2/STAT3 signaling pathway in mice during sevoflurane anesthesia" was retracted in 2021. Reasons: duplicated images; signs of a paper mill.

Our data further revealed that *miR-135b-5p* inhibition improved cardioprotective functioning of sevoflurane by activating the JAK2/STAT3 signaling pathway. MiRNAs have been recognized to be a crucial regulator in a number of diseases including human cancers, immunological disorders as well as cardiovascular diseases [22–24]. Some miRNAs have been reported in myocardial I/R injury [25,26]. *MiR-135* inhibitors can contribute to the induction of myogenic differentiation of dental pulp stem cells [27]. Importantly, *miR-135b* once was involved in cancer growth [28], invasiveness [29], and motility [30], and it was up-regulated in various other tumor types, including colon, breast, lung, and prostate tumors [29,31,32]. Interestingly, *miR-135b* function has been adapted and treated as an oncogenic biomarker [29,30]. Thus, so far, four mammalian JAKs and seven mammalian STATs have been identified [20]. The JAK2/STAT3 pathway is highly evolutionarily conserved and participates in growth and development, intercellular communication, signaling transduction, and gene transcription [33]. In recent years, various studies have demonstrated that the JAK2/STAT3 signal pathway is activated in cellular and animal models of I/R injury including models of heart I/R injury, revealing an important role of JAK2/STAT3 signaling pathway in the regulation of I/R injury [34,35]. We also confirmed that JAK2 was the target gene of *miR-135b-5p*. Thus, we conclude that *miR-135b-5p* could mediate the cardioprotective functioning of sevoflurane by up-regulating JAK2 expression.

In our experiment, in comparison with the Sevo and inhibitor + AG490 + Sevo groups, the AG490 + Sevo group showed decreased LVEF, LVFS, Bcl-2 expression, mRNA expression of JAK2 and STAT3, and protein expression of p-STAT3 and p-JAK2, but increased cardiomyocyte necrosis, apoptosis, and Bax expression, while opposite trends were seen in the inhibitor + Sevo group. Bax is commonly adapted as a pro-apoptotic protein, while Bcl-2 is often regarded as an anti-apoptotic protein [36]. Additionally, one indirect model demonstrates that Bax activation cannot be achieved if all anti-apoptotic Bcl-2 proteins are neutralized [37]. Current principle for pivotal restriction for sudden cardiac death has adapted a LVEF no more than 35% as a critical point in patients who displayed nonischemic dilated cardiomyopathy and post-myocardial infarction [38]. The research of Tian et al. [33] shows that ischemia postconditioning may attenuate myocardial apoptosis in the process of prolonged reperfusion by regulating JAK2/STAT3/Bcl-2 pathway. Some cardioprotective agents such as fasudil are capable of protecting myocardial tissues against I/R injury by activating the JAK2/STAT3 signaling pathway [39]. The study of Kim et al. [40] demonstrates that sevoflurane postconditioning decreases apoptosis by up-regulating p-JAK, p-STAT, and Bcl-2 expression and decreasing Bax expression after transient global ischemia in rats, and once JAK2 was inhibited, the anti-apoptotic effects of sevoflurane were reversed, suggesting that the JAK2-STAT3 pathway may be associated with the anti-apoptotic functioning of sevoflurane postconditioning. All data above were in-line with our findings, thus, we conclude that inhibition of *miR-135b-5p* could enhance myocardial I/R injury by elevating JAK2 expression and activating the JAK2/STAT3 signaling pathway.

The article "Suppression of microRNA-135b-5p protects against myocardial ischemia/reperfusion injury by activating JAK2/STAT3 signaling pathway in mice during sevoflurane anesthesia" was retracted in 2021. Reasons: duplicated images; signs of a paper mill.

## Conclusion

To conclude, our study provided evidence that *miR-135b-5p* inhibition could enhance JAK2 expression, activate JAK2/STAT3 signaling pathway, contributing to the protection of myocardial I/R injury. The present study sheds new light on the molecular mechanisms whereby miRNAs might participate in the myocardial I/R injury, which provides novel evidence for I/R injury management.

## Abbreviations

AI: apoptotic index
Bax: Bcl-2 associated X protein B
Bcl-2: B-cell lymphoma-2
DMEM: Dulbecco’s modified Eagle’s medium
ECG: electrocardiogram
HE: hematoxylin-eosin
HIF-1alpha: hypoxia-inducible factor 1 alpha
I/R: ischemia/reperfusion
JAK: Janus protein tyrosine kinase
LVDD: left ventricular end-diastolic diameter
LVDV: left ventricular end-diastolic volume
LVEF: left ventricular ejection fraction
LVSD: left ventricular end-systolic diameter
LVSV: left ventricular end-systolic volume
mut: mutation
NOS: nitricoxide synthase
qRT-PCR: quantitative real-time PCR
Sevo: sevoflurane
STAT: signal transducer and activator of transcription
TBST: tris-buffered saline Tween-20
TUNEL: terminal dexynucleotidyl transferase mediated dUTP-biotin nick end labeling
wt: wild-type
